The article "Comparison of Minimally Invasive Surgery Transforaminal Lumbar Interbody Fusion and TLIF for Treatment of Lumbar Spine Stenosis" was published in 2022. Journal: J Healthc Eng.

# Comparison of Minimally Invasive Surgery Transforaminal Lumbar Interbody Fusion and TLIF for Treatment of Lumbar Spine Stenosis

**DOI:** 10.1155/2022/9389239

**Published:** 2022-01-25

**Authors:** Guodong Gao, Linzhong Cao, Xiaozheng Du, Bin Xu, Ping Zhang, Xiaogang Zhang, Rong Wang, Zhen Quan

**Affiliations:** ^1^Department of Spinal Surgery, Affiliated Hospital of Gansu University of Chinese Medicine, Gansu 730000, China; ^2^College of Electrical and Information Engineering, Lanzhou University of Technology, Gansu 730050, China

## Abstract

With the development of minimally invasive technology, minimally invasive surgery transforaminal lumbar interbody fusion has become an effective way to treat lumbar spinal stenosis. Lumbar spinal stenosis is one of the common diseases that cause backache or lumbago and sciatica. This article compares and analyzes the clinical efficacy of 60 patients with lumbar spinal stenosis surgery. It can be seen that the wound by MIS-TLIF is significantly less than that of traditional open surgery, and the postoperative recovery of MIS-TLIF is faster. So, MIS-TLIF is one of the concepts of minimally invasive surgery. The age distribution ranged from 56 to 78 years, with an average of 65.7 years. 31 cases were treated with MIS-TLIF (MIS-TLIF group), and 29 were treated with traditional posterior open surgery (TLIF group). The operation time, intraoperative blood loss, and postoperative drainage of the operation area were recorded. After statistical testing, the intraoperative blood loss, incision size, and postoperative drainage volume of the wound in the MIS-TLIF group were significantly less than those in the TLIF group. The results of JOA score, ODI score, and VAS score during the postoperative follow-up period were comparable to those of open surgery. Therefore, minimally invasive transforaminal lumbar interbody fusion is effective in treating lumbar spinal stenosis.

## 1. Introduction

Lumbar spinal stenosis is a degenerative disease of the spine related to labor intensity and lumbar load. It is caused by the proliferation and hypertrophy of the ligamentum flavum, the proliferation and cohesion of the facet joints, the degeneration of the intervertebral disc, and the degeneration of the lumbar spine [1, 2]. The reduced diameter of the canal, lateral recess, and nerve root canal causes the volume of the spinal canal to decrease and nerve root compression and corresponding neurological dysfunction. It is also a common clinical disease and frequently occurring disease that causes low back pain or low back pain. Its main clinical features are neurological intermittent claudication, as well as weakness and discomfort of the buttocks, thighs, and calves, which aggravate after walking or extension. Another clinical feature is paraesthesia in the sellar area (perineum) and abnormal bowel function. In clinical practice, the disease is mostly treated with surgery, and traditional surgery is mostly with open transforaminal lumbar fusion [3, 4]. However, during the implementation of open surgery, there are problems such as large surgical incisions, damage to the muscle anchor point, large traction damage, excessive intraoperative bleeding, postoperative soft tissue scarring, muscle atrophy, high infection rate, and long hospital stay. With the continuous deepening of the concept and technology of minimally invasive surgery, MIS-TLIF is due to its significantly reduced access-related complications, small soft-tissue damage, less surgical blood loss, light postoperative pain, early getting out of bed, quick recovery, and short hospital stay And other advantages are getting more and more recognition from doctors and patients [5, 6].

The article "Comparison of Minimally Invasive Surgery Transforaminal Lumbar Interbody Fusion and TLIF for Treatment of Lumbar Spine Stenosis" was published in 2022. Journal: J Healthc Eng.

There are about 300 lumbar minimally invasive patients in our hospital every year, and all patients did not respond to conservative treatment. This article selects 60 patients with lumbar spinal stenosis who were treated in our hospital from September 2019 to March 2021 as the research object to compare the clinical effects of minimally invasive transforaminal lumbar interbody fusion and open TLIF surgery. In order to ensure the curative effect, different surgical methods were used to different patient.

The rest of this paper is organized as follows.  Section 2 discusses the patients and methods of operation, followed by the typical cases from 60 patients in Section 3. Comparison of curative effect between two groups is discussed in Section 4.  Section 5 concludes the paper with summary and future research directions.

## 2. Patients and Methods of Operation

### 2.1. General Information

Sixty patients with lumbar spinal stenosis who were treated in our hospital from April 2019 to August 2020 were selected as the research objects. The general statistics of the patients are shown in Table 1. Among them, there were 24 males and 36 females; the age ranged from 56 to 78 years, with an average of 65.7 years; the course of illness was from 6 to 128 months, with an average of 12.6 months. Most cases had recurrent clinical symptoms and were admitted to the hospital due to recent worsening. Among them, 54 cases (90%) were low back pain, 23 cases (38.3%) were neurological intermittent claudication of both lower limbs, and 37 cases (61.7%) were unilateral nerve root pain and/or numbness. Patients' signs were as follows: 43 cases (71.5%) of lower extremity sensory function abnormality, 21 cases (35%) of lower extremity motor function abnormality, 8 cases (13.3%) of tendon reflexes, and 13 cases (21.7%) of the straight leg elevation test were positive. All selected patients were diagnosed with lumbar spinal stenosis through clinical symptoms and imaging examinations, and patients with severe heart, kidney, liver, and other important organ dysfunction and severe mental illness were excluded. Among them, 31 patients underwent MIS-TLIF surgery and were set as MIS-TLIF group; 29 patients underwent TLIF surgery and were set as TLIF group. The two groups of patients have no statistical difference in general information such as age, gender, course of disease, weight, onset nerve segment, and symptoms, and they are comparable (*P* > 0.05).

The article "Comparison of Minimally Invasive Surgery Transforaminal Lumbar Interbody Fusion and TLIF for Treatment of Lumbar Spine Stenosis" was published in 2022. Journal: J Healthc Eng.

### 2.2. Surgical Methods of TLIF

The patient was under general anesthesia, routinely sterilized, and draped in a prone position, with the abdomen hanging in the air Take the level of the intervertebral disc of the adjacent vertebral body as the center; make a median longitudinal skin incision, about 8–10 cm long, to expose the spinous process of the diseased segment, the upper and lower facet joints, and the lamina of the lower vertebrae, with the transverse process. The intersection of the midline and the outer edge of the articular process is the needle entry point, and the positioning needle is placed on both sides, and the pedicle screw is inserted after the fluoroscopy is correct. Then, use a bone knife to cut off the inferior articular process on one side of the diseased segment, and then cut off the medial and upper edge of the upper articular process (decompression bone treatment is small granular for spare intervertebral bone grafting), and open the intervertebral foramen. After decompression, bite off the ligamentum flavum, expose the dural sac, expand the nerve root canal, fully expose and loosen the nerve root, thoroughly remove the intervertebral disc and cartilage endplate, flush the intervertebral space, and fill the front of the intervertebral space with autologous decompression bone particles. Place a suitable intervertebral fusion cage. If it is bilateral symptoms, the same ascending bilateral decompression, then place the connecting rods on both sides and lock them up after proper opposing pressure. The patient was fluoroscoped again and again to determine the internal fixation position. Thoroughly stop bleeding and flush the incision, place a drainage tube on the incision, and suture layer by layer.

### 2.3. Surgical Methods of MIS-TLIF

The patient was under general anesthesia, routinely sterilized drapes, and prone position. Under C-arm X-ray machine fluoroscopy, the projection point of the pedicle body surface of the surgical segment was marked. Make a lateral central skin incision of about 3.5 cm at the posterior midline of the affected side from 2.5 to 3.0 cm (depending on the diseased segment and patient size). Cut the skin, subcutaneous tissue, and deep fascia layer by layer, with more blunt separations. A step-by-step dilation tube is placed between the fission muscle and the longissimus muscle to establish a quadrant working channel, and the free arm is fixed. Expose the facet joints, insert a positioning needle 2 mm inward and downward from the root of the transverse process, and perform decompression after the fluoroscopy is correct.

The article "Comparison of Minimally Invasive Surgery Transforaminal Lumbar Interbody Fusion and TLIF for Treatment of Lumbar Spine Stenosis" was published in 2022. Journal: J Healthc Eng.

*Bilateral Decompression of the Bilateral Approach.* First, remove most of the lower and upper articular processes on the side with mild symptoms, bite off the lamina to the root of the spinous process on the dorsal side of the ligamentum flavum, and then remove the ligamentum flavum. Fully loosen the dural sac and nerve roots. Then, place the pedicle screw and place the connecting rod to lock the intervertebral space after proper compression; then replace the working channel on the side with more severe symptoms, perform spinal decompression in the same way, reveal the triangle of Kambin, and gradually expand the intervertebral space. Fully remove the intervertebral disc tissue. A bone grafting funnel is used to fill the front of the intervertebral space with autogenous decompression bone particles and place a suitable intervertebral fusion cage. Place the pedicle screw and place the connecting rod to lock up after proper compression [7, 8].

### 2.4. Observation Index and Efficacy Judgment

The surgical efficacy of the two groups of patients was compared, and the operation time, intraoperative blood loss, bed time, postoperative blood transfusion, postoperative drainage volume, and other surgical indicators were compared between the two groups. The two groups were compared 1 day before and 6 months after surgery. *Clinical Symptoms.* The overall condition of the patient was evaluated by the JOA score, which is the curative effect evaluation standard of the Japanese Orthopedic Branch, the visual analogue score VAS was used to evaluate the patient's waist and leg pain, and the Oswestry Disability Index (ODI) was used to evaluate the patient's waist function. The incidence of adverse reactions such as postoperative infection, nerve root injury, hard sac rupture, and the total incidence of adverse reactions were compared between the two groups. The Prolo functional evaluation standard after lumbar fusion was used to evaluate the surgical efficacy of patients, including two parts: functional score and symptom score. Among them were recovery: total score of 8–10; effective total score of 6–7; and invalid: total score of 5 and 5 points or less [9, 10].

The article "Comparison of Minimally Invasive Surgery Transforaminal Lumbar Interbody Fusion and TLIF for Treatment of Lumbar Spine Stenosis" was published in 2022. Journal: J Healthc Eng.

Observe and compare the two groups' operation time, incision size, intraoperative blood loss, hospital stay, time spent on the ground, and other indicators. At the same time, observe and compare the pain index of the two groups at 1, 3, and 6 months after surgery, according to the visual analog scale of pain (VAS). The assessment was as follows: 0 points are painless as 0 grade, 1–3 are divided into (i) grade, 4–6 are divided into (ii) grade, 7–10 are divided into (iii) grade; the higher the score, the more severe the pain [11, 12].

The functional recovery is evaluated according to the scores of the Japanese Orthopedic Association (JOA), which mainly include subjective symptoms (9 points), clinical signs (6 points), and daily life limitations (14 points). The higher the score for each item, the better the functional recovery.

### 2.5. Statistical Analysis

In this study, SPSS 22.0 statistical software was used to analyze the data. The measurement data was expressed as the mean ± standard deviation ($\tilde{\text{x}}\pm \text{s}$). The *t*-test was used for comparison between two groups; the *γ*^2^-test was used for comparison between two groups. The difference was statistically significant (*P* < 0.05).

## 3. Typical Cases

### 3.1. Case 1

In this case, Liu is a 72-year-old woman and she is sick with L4-5 single space spinal stenosis. Related image data before and after surgery are shown in Figure 1. The patient's lumbar hyperplasia stenosis was so severe that surgical treatment used is bilateral approach and bilateral decompression method.

Surgical treatment used is bilateral approach and bilateral decompression method. Figure 1(a) is preoperative MRI of sagittal view. Figure 1(b) is preoperative MRI of shaft position. Figure 1(c) is preoperative CT of axis position. Figure 1(d) is the intraoperative C-arm positioning and placement of channel. Figure 1(e) is frontal X-ray in 1 month after operation. Figure 1(f) is lateral X-ray in 1 month after operation.

### 3.2. Case 2

In this case, Shi is a 69-year-old woman and she is sick with double-space spinal stenosis. Related image data before and after surgery are shown in Figure 2. Surgical treatment is used unilateral approach unilateral double gap decompression method. The specific operation is using spinal canal decompression, intervertebral space treatment, and cage placement and dural sac nerve root decompression only in symptom side. And then, placement of the pedicle screws pass through the Wiltse at the contralateral channel.

The article "Comparison of Minimally Invasive Surgery Transforaminal Lumbar Interbody Fusion and TLIF for Treatment of Lumbar Spine Stenosis" was published in 2022. Journal: J Healthc Eng.

Figure 2(a) preoperative MRI of sagittal view. Figure 2(b) is the preoperative CT in axis position. Figure 2(c) is the postoperative CT in axis position. Figure 2(d) is postoperative MRI at shaft position and muscle injury. Figure 2(e) is the postoperative CT of intervertebral bone graft fusion. Figure 2(f) is frontal X-ray in 1 month after operation. Figure 2(g) is lateral X-ray in 1 month after operation.

### 3.3. Case 3

In this case, Zhao is a 48-year-old woman and she is sick with prolapse of nucleus pulposus of lumbar spine and Modic changes in intervertebral space. Related image data before and after surgery are shown in Figure 3. Surgical MIS-TLIF treatment is used to patient which of through the VISTA channel with microscope.

Figure 3(a) is preoperative MRI of sagittal view. Figure 3(b) is message of decompression in progress at the operation. Figure 3(c) is message of channel in progress at the operation. Figure 3(d) is the postoperative CT of intervertebral bone graft fusion. Figure 3(e) is the postoperative MRI in 3 months after operation. Figure 3(f) is frontal X-ray in 1 month after operation. Figure 3(g) is lateral X-ray in 1 month after operation. Figure 3(h) is CT in 7 months after operation. From all of the messages, we can get the following conclusion that the bone of lumbar spine is fusion.

### 3.4. Case 4

In this case, Chen is a 75-year-old woman and she is sick with straitness of lumbar vertebrae at L4/5. Related image data before and after surgery are shown in Figure 4. Surgical MIS-TLIF treatment is used to patient which of through the VISTA channel with microscope. Figure 4(a) is preoperative CT of sagittal view. It can be obtained from the figure that the patient has severe spinal stenosis in L4/5 and ossification at ligamentum flavum. Figure 4(b) is preoperative MRI of sagittal view. Figure 4(c) is the preoperative CT at shaft position. Figure 4(d) is the postoperative CT at shaft position. Figure 4(e) is meninx fibrosa and nerve root at postoperative period.

Figure 4(f) is postoperative MRI at shaft position and muscle injury. Figure 4(g) is lateral position X-ray in 1 month after operation. It indicates that the nail position is well fixed, and the position of the fusion device is well implanted. Figure 4(h) is frontal X-ray in 1 month after operation. Figure 4(i) is transverse incision.

### 3.5. Case 5

In this case, Wang is a 65-year-old woman and she is sick with adult degenerative scoliosis with double-segmental stenosis. Related image data before and after surgery are shown in Figure 5. MIS-TLIF treatment is done to the patient. Figure 5(a) is preoperative MRI of sagittal view. Figure 5(b) is preoperative CT of the coronal view. Figure 5(c) is the preoperative MRI at shaft position at L3/4. Figure 5(d) is the postoperative MRI at shaft position at L3/4. Figure 5(e) is the preoperative MRI at shaft position at L4/5. Figure 5(f) is the postoperative MRI at shaft position at L4/5.

The article "Comparison of Minimally Invasive Surgery Transforaminal Lumbar Interbody Fusion and TLIF for Treatment of Lumbar Spine Stenosis" was published in 2022. Journal: J Healthc Eng.

Figure 5(g) is frontal X-ray in 1 month after operation. Figure 5(h) is lateral position X-ray in 1 month after operation. Figure 5(i) is anteroposterior X-ray of the patient's spine one year after surgery. Figure 5(j) is lateral X-ray of the patient's spine one year after surgery. From Figures 5(i) and 5(j), it can be seen from the figure that the coronal and sagittal positions of the spine are balanced. Figure 5(k) is transverse incision.

## 4. Analysis of MIS⁃TLIF and TLIF

### 4.1. Comparison of the Advantages and Disadvantages of MIS-TLIF and TLIF

The comparison of surgical efficacy between the MIS-TLIF group and the TLIF group is shown in Table 2. It can be seen that the recovery rate and total effective rate after surgery in the MIS-TLIF group were significantly higher than those in the TLIF group, and the difference was statistically significant (*P* < 0.05). There was no significant difference in the effective rate after surgery between the two groups, *P* > 0.05.

The relevant data of patients in the MIS-TLIF group and TLIF group during the perioperative period are shown in Table 3. Compared with the TLIF group, the MIS-TLIF group has a longer operation time, a small surgical incision, a significant reduction in intraoperative blood loss, a 37.7% reduction in postoperative drainage, and a 32.3% and 13.9% reduction in hospital stay and hospital costs, respectively.

Comparison of all of clinical symptoms between the two groups of patients during 1 year after surgery: during the follow-up period, no complications such as infection, internal fixation, and fusion failure were occurred. At the last follow-up, the pain score was evaluated according to the pain visual analogue scale (VAS). The results are shown in Table 4. The pain level of the two groups of patients after surgery decreased. The VAS of the patients in the MIS-TLIF group at 2, 5, and 12 months after surgery: the scores were all lower than the TLIF group; the difference was statistically significant (*P* < 0.05).

The JOA scores of the two groups of patients at 6 months after operation are shown in Table 5. The subjective symptom score of the MIS-TLIF group was significantly higher than that of the TLIF group; the difference was statistically significant (*P* < 0.05); the clinical symptom score of the MIS-TLIF group was significantly higher than that of the TLIF group. In the TLIF group, the difference was statistically significant (*P* < 0.05); the daily activity ability score of the MIS-TLIF group was significantly higher than that of the TLIF group, and the difference was statistically significant (*P* < 0.05).

The article "Comparison of Minimally Invasive Surgery Transforaminal Lumbar Interbody Fusion and TLIF for Treatment of Lumbar Spine Stenosis" was published in 2022. Journal: J Healthc Eng.

MIS-TLIF better preserves the lumbar spinous process, interspinous ligament, and local blood supply of the psoas muscle, which is more conducive to the recovery of patients after surgery. In MIS-TLIF, by moving the working channel inward, the decompression range is expanded, and effective decompression can also be performed for part of the lumbar central canal stenosis [13, 14]. It also avoids stripping and excessive stretching of the paraspinal muscles on both sides, retains the structural function of the posterior tension band of the lumbar spine, increases the biomechanical stability of the spine, and effectively reduces the formation of low back muscle atrophy and soft tissue scars, which is beneficial to the recovery of back muscle function reduces the incidence of low back pain after surgery, shortens the time for patients to go to the ground, and also reduces the economic burden of patients.

So, MIS⁃TLIF has some advantages as follows: it has fewer concomitant symptom after the surgery, the patient's pain is minor and relieved, soft tissue damage of the patient is minimal, and the patients have a short recovery time. On the other side, MIS⁃TLIF has some disadvantages as follows: the operation time is long, the cost of internal fixation is high, and the surgical operator must have great skill.

### 4.2. Analysis of the Safety and Effectiveness of MIS-TLIF

Regarding the stability of bone graft fusion, the MIS-TLIF group used a bone knife during decompression to appropriately resect the lamina in the direction of the spinous process root, treat the decompressed bone, and then implant it into the intervertebral space. The amount of bone graft was equivalent to that of the TLIF group. It is possible to place an intervertebral fusion cage obliquely into the intervertebral space without using allogeneic bone or BMP. With the aid of pedicle screws, the effect of shearing force is eliminated and the bone graft fusion rate is improved.

One case of early infection is found from 31 patients in the MIS-TLIF group and the details are as follows. The patient developed high fever and chills on the 9th day after surgery. After rechecking the inflammatory index, postoperative complications were repeated hemorrhages. After the second debridement, vancomycin bone cement was used in patient. The fever gradually disappeared after the operation, and the local back pain was significantly relieved. After two weeks, the wound was healed and the sutures were removed. Three months later, the patient walked freely. The cause of infection was analyzed after surgery. The patient was treated with radiotherapy and chemotherapy almost one year after right breast cancer resection. The body immunity was low. On the other hand, the patient was allergic to cephalosporin antibiotics. Clindamycin was used for 2 days after surgery.

The article "Comparison of Minimally Invasive Surgery Transforaminal Lumbar Interbody Fusion and TLIF for Treatment of Lumbar Spine Stenosis" was published in 2022. Journal: J Healthc Eng.

There was 1 case of dura damage form the MIS-TLIF group. The location was close to the dorsal side of the exit root. It was temporarily compressed by gelatin sponge and cotton pads to complete the intervertebral space treatment and nerve root decompression as soon as possible; then, it was washed by a large amount of saline. When the cotton was removed, gelatin sponge was applied for compression. After the operation, it was found that the drainage volume did not increase significantly, so the drainage tube was removed normally. No complications related to dura damage were seen after the operation.

Despite the above, the functional scores of patients in the MIS-TLIF group are still significantly higher than those of the TLIF group. On the whole, the treatment effect of the MIS-TLIF group is better than that of the TLIF group (*P* < 0.05), indicating that the minimally invasive transvertebral foraminal lumbar interbody fusion can improve the treatment effect. The posterior vertebral body fusion will damage the soft tissue of the back of the lumbar spine relatively, and the postoperative complication rate is relatively high, which delays the speed of postoperative physical recovery [15].

Compared with TLIF, MIS-TILF can achieve sufficient and effective decompression, reconstruction of lumbar spine sequence and stability, reduce surgical trauma, shorten the time spent in bed, and accelerate the postoperative spinal function recovery of patients. Through the comparative analysis of MIS-TLIF, we can better master this technology for its analysis and research.

## 5. Conclusion

In recent years, with the continuous improvement of living standards, people's material living standards have been significantly improved, and the requirements for medical methods have also been continuously improved. In the clinical treatment of lumbar spinal stenosis, open posterior vertebral body fusion is widely used, but due to the large surgical trauma, heavy bleeding, and large postoperative drainage, it is easy to affect postoperative physical recovery. Minimally invasive transforaminal lumbar interbody fusion for the treatment of lumbar spinal stenosis has received more and more attention from doctors and patients because of its advantages such as less soft tissue damage, less blood loss, and faster recovery after surgery.

The article "Comparison of Minimally Invasive Surgery Transforaminal Lumbar Interbody Fusion and TLIF for Treatment of Lumbar Spine Stenosis" was published in 2022. Journal: J Healthc Eng.

In summary, MIS-TILF and TILF surgery can clearly improve the symptoms of patients with lumbar spinal stenosis, and the clinical effect is significant. Compared with TILF surgery, MIS-TILF has the advantages of less damage to muscle and nerve tissue, less intraoperative bleeding, and faster postoperative recovery. With the development of minimally invasive spinal surgery, MIS-TILF will be more widely used in the treatment of lumbar degenerative diseases through continuous summary and improvement.

## Figures and Tables

**Figure 1:** Treatment information of case 1.

**Figure 2:** Treatment information of case 2.

**Figure 3:** Treatment information of case 3.

**Figure 4:** Treatment information of case 4.

**Figure 5:** Treatment information of case 5.

**Table 1:** Patients' information statistics.

Groups	Instance data	Gender		Weight (kg)	Mean disease course (months)	Onset of segment		
		Male	Female			L4-5	L5-S1	L4-S1
MIS⁃TLIF	30	12	19	67.13	12.7	16	10	5
TLIF	30	13	16	66.97	12.5	14	9	6

^*∗*^The general data between the two groups were insignificant and comparable（*P* > 0.05）.

**Table 2:** Comparison of surgical efficacy between two groups of patients （*n*, %）.

Groups	Instance data	Recovery	Effective	Invalid	Total effective rate
MIS⁃TLIF	31	26 (83.9)	5 (16.1)	0 (0)	31 (100)
TLIF	29	22 (75.9)	7 (24.1)	00 (0)	29 (100)
*γ* ^2^					4.32
*P*					<0.05

**Table 3:** Perioperative data and comparison of the two groups of patients.

Groups	Instance data	Mean length of wds (cm)	Mean operating time (h)	Mean intraoperative blood loss (mL)	Mean postoperative drainage volume (mL)	Average hospital costs/ten thousand yuan	Mean postoperative exercise time (d)/d	Average stay (d)
MIS⁃TLIF	31	3.4	2.6	127.6	98.8	3.1	3.5	8.2
TLIF	29	8.5	2.2	187.4	29 (100)	3.6	5.8	12.1

**Table 4:** VAS score and comparison table at different time points after the operation of the two groups.

Groups	Instance data	2 months after surgery	Five months after surgery	12 months after surgery
MIS⁃TLIF	31	3.12 ± 1.01	1.63 ± 0.81	1.58 ± 0.61
TLIF	29	4.52 ± 1.32	2.62 ± 1.09	1.72 ± 0.89
*t*		5.32	5.89	3.12
*P*		<0.001	<0.001	<0.004

**Table 5:** Results and comparison of JOA scores for the last follow-up in the two groups.

Groups	Instance data	Subjective symptom	Clinical symptoms	Daily activity ability
MIS⁃TLIF	31	7.71 ± 1.29	5.43 ± 0.61	12.39 ± 1.61
TLIF	29	5.42 ± 1.47	3.42 ± 0.81	10.78 ± 1.59
*t*		7.86	15.01	4.11
*P*		<0.001	<0.001	<0.001

## Data Availability

The medical data and figure used to support the findings of this study are available from the corresponding author upon request.
